# Influence of Heat Stress on Intestinal Epithelial Barrier Function, Tight Junction Protein, and Immune and Reproductive Physiology

**DOI:** 10.1155/2022/8547379

**Published:** 2022-09-01

**Authors:** Sahar Ghulam Mohyuddin, Imran Khan, Ahmad Zada, Aftab Qamar, Abdelaziz Adam Idriss Arbab, Xin-bing Ma, Zhi-chao Yu, Xiao-Xi Liu, Yan-Hong Yong, Xiang Hong Ju, Yang Zhang-Ping, Mao Yong Jiang

**Affiliations:** ^1^College of Animal Science and Technology, Yangzhou University, Yangzhou 225009, China; ^2^Department of Animal Science, College of Coastal Agricultural Sciences, Guangdong Ocean University, Zhanjiang, Guangdong 524088, China; ^3^College of Bioscience and Biotechnology, Yangzhou University, Yangzhou 225009, China; ^4^Department of Veterinary Medicine, College of Coastal Agricultural Sciences, Guangdong Ocean University, Zhanjiang, Guangdong 524088, China

## Abstract

The potential threat of global warming in the 21^st^ century is on the ecosystem through many aspects, including the negative impact of rising global temperature on the health of humans and animals, especially domestic animals. The damage caused by heat stress to animals has been more and more significant as the worldwide climate continues to rise, along with the breeding industry's expanding scale and stocking density, and it has become the most important stress-causing factor in southern China. In this review, we described the effects of heat stress on animal immune organs and immune system. The much-debated topic is how hyperthermia affects the tight junction barrier. Heat stress also induces inflammation in the body of animals causing low body weight and loss of appetite. This review also discussed that heat stress leads to hepatic disorder, and it also damages the intestine. The small intestine experiences ischemia, and the permeability of the intestine increases. Furthermore, the oxidative stress and mitogen-activated protein kinase (MAPK) pathways have a significant role in stress-induced cellular and organ injury. The study has shown that MAPK activity in the small intestine was increased by heat stress. Heat stress caused extreme small intestine damage, enhanced oxidative stress, and activated MAPK signaling pathways.

## 1. Introduction

The global temperature is increasing day by day, and this change affects all living organisms on earth. An increase in temperature is very harmful to humans and animal growth, production, and health. Elevated temperature in the circumstance of global warming is likely to affect life on earth adversely. Excessive heat load makes animals more susceptible to multiple diseases compromising the functioning of different immune system components. Heat stress produces significant economic losses in the livestock sector as it severely compromises farm animal productivity. The body temperature of animals increased in response to high environmental temperature. Heat stress has a negative impact on an animal's normal physiological functioning, and it appears when the body is unable to lose heat by physiological mechanisms [1]. The effects of heat stress on animals depend upon the time frequency of heat exposure [2]. Long-term heat exposure causes changes in the physiology of animals; it also damages the body system of animals [3]. In contrast, short-term heat exposure causes tissue damage and fast synthesis of heat shock proteins, which plays an essential role in regulating short-term and long-term heat exposure.

Heat stress leads to physical and behavioral changes in the body. Variations in environmental factors like temperature, sunlight, humidity, and changes in animal metabolism may lead to abnormal body responses [4]. Long-term exposure to heat may cause severe damage to immune responses and endocrine, cardiovascular, and respiratory system disorders. The negative effect of heat stress on domestic livestock and poultry may include decreased production rate, milk yield, and reproductive efficiency and reduced egg yield. Heat stress is a cause of oxidative stress in summer in domestic animals [5]. Many researchers have observed that under heat stress, the concentration of reactive oxygen species (ROS) increases and leads to oxidative damage in the body [6].

The gastrointestinal tract acts as a physical barrier against toxic substances and thus protects the internal environment from harmful objects. It could be possible by the protein harmonization process in the cell to cell connection, such as tight junctions [7]. The tight junction is a complicated system that maintains the transport of ions, molecules, and water. Transmembrane proteins include occludin, claudin, tricellulin, and junctional adhesion molecule (JAM). Most researchers have described that tight junction permeability and tight junction protein expression/cytoskeleton are maintained through signaling pathways such as MAPK, PKC, and PI3K and protein phosphatases [8]. Disruption of the epithelial barrier in the gut allows molecules in the intestinal lumen as well as opportunistic/pathogenic microbiota and the entrance to gut-associated immune organs and elicits an inflammatory response. Most researchers have described that proinflammatory cytokines like TNF-*α*, INF-*γ*, IL-1*β*, and IL-13 decrease barriers by reducing the expression of tight junction proteins and stimulating epithelial apoptosis. The alteration in cytokines and their outcomes related to the tight junction during the inflammation process is complex and needs more exploration [9].

Moreover, in another research, pregnancy and lactating retrospectives of animals are more affected by heat stress [10]. Heat stress interferes with normal animal performance. The effect of heat stress has been reported in human beings [11], domestic animals [12], pigs [13, 14], and rodents [15, 16].

## 2. Stress

Stress has no specific definition [13]. Stress is a neuroendocrine response of the body, triggered by internal or external stimuli, in order to adapt to a specific condition, e.g., heat, and establish homeostasis. Stress is the response of the animal to a specific condition. The body does not combat stress; the body uses stress as a response to a condition and by this response looks for an adaptation. In a stressed situation, the animal's body automatically responds to combat the negative effect of stress. Stress changes the body inner temperature by disturbing its thermoregulatory mechanisms. Stress can be of two categories, specific or nonspecific. It has three phases: (1) fear is called an alarm; (2) when the body resists the environmental change, then it is called resistance [13]; and (3) when the temperature increases beyond the limits, the body does not tolerate the change and is called exhaustion [14, 15].

Moreover, heat stress is also a cause of disruption between anti- and proinflammatory cytokines [16]. Many studies have reported the effects of heat stress on humans [17] and animal models [18]. The increased number of free radicals and inflammatory cytokines and reduced amount of antioxidant that causes disorder in the liver has also been observed. Due to heat stress, small intestine ischemia is also a contributing factor in the production of reactive oxygen species [19].

### 2.1. Mechanism of Heat Stress

The time and severity of heat are the main drivers that produce the effect on an animal body. A study has described that in heat stress, the animal eats less but drinks more, is drowsy most of the time, is reluctant to move, and raises. In maintaining body homeostasis, the neuroendocrine system plays a crucial role in controlling the unfavorable effects. During heat stress, the neuroendocrine system is activated, which stimulates the sympathetic-adrenal medullar axis with the hypothalamic-pituitary adrenal axis [20], leading to the production of glucose in the body of the mouse [21].

The hypothalamus-pituitary-adrenal (HPA) axis is the primary indicator, identifier, and control point of stress [22]. Adrenocorticotropic hormone (ACTH) is the HPA axis product that controls heat stress in the body. It also controls the synthesis and release of cortisol. During stress conditions, the adrenal gland will produce aldosterone to regulate the electrolyte balance [19]. ACTH and HPA axis released corticosterone, and it has a slow release rate but long-lasting effects during heat stress [23], while a higher concentration of secreting corticosterone may result in heart problems, decreased immunity, and mental stress [24]. Studies have shown that heat stress affects the reproductive system of the animal as it reduces the activity of hormones involved in sexual function. Studies have shown that the mouse immune system gets disturbed at a high temperature due to the abnormal production of cytokines [25]. Studies have shown that heat stress has a negative influence on various chicken species, including lower growth rates, appetites, feed consumption, and laying, as well as compromised meat and egg quality.

Interleukin 6 (IL-6) is a pleiotropic cytokine that is important in most disease conditions. IL-6 secretions will be automatically enhanced in animals that suffer from diseases. Typically, during intestinal inflammation, it is produced in large amounts. It is reported that IL-6 increases the expression of channel-forming claudin-2, which is important for caudal-related MEK/ERK and P13K pathways in intestinal epithelial cells. It has been reported that different pathways are concerned with tight junction permeability and claudin-2 expression through IL-6 [26]. The communication between the nervous and immune systems is shown in Figure 1.

### 2.2. Heat Stress and (HPA) Axis Pathway

The HPA axis plays a vital role in the secretions of many neurotransmitters and hormones important in animal thermoregulation. Glucocorticoids, adrenocorticotropin-releasing hormone, and corticotropin-releasing factors that maintain hyperthermia pathways in animals are released from the HPA axis. Corticotropin-releasing factor (CRF) is produced and released from the paraventricular nucleus of the hypothalamus. It controls the HPA axis during heat stress. CRF causes the release of adrenocorticotropic hormone (ACTH) from the anterior pituitary [27]. When CRF gets attached to the receptor, ACTH begins to be released in the circulation [28]. As a result, glucocorticoid begins to release and regulate the effect of change due to high temperature. The adrenal gland is the main site for circulating ACTH, where it triggers glucocorticoid production and secretions from the zona fasciculate. Glucocorticoids play the role of downstream effectors for the HPA axis; in intracellular receptors, they produce alteration for the maintenance of physiological processes [29]. Under extreme circumstances, glucocorticoids play an important role in coping with unusual circumstances. But the HPA axis and health of animals might be affected by the degree of production and release of glucocorticoids [30]. Cortisol plays a significant role in regulating the physiological processes; it increases food requirements, thus increasing the availability of glucose and depressing another system of the animal body [31].

### 2.3. Impact of Heat Stress on Animal Performance

Heat stress refers to the sum of a series of nonspecific physiological responses exhibited by an animal to a heat source in an extremely high-temperature environment. The difference in stress intensity and stress time has a great impact on the health of the body. Mild and short-term heat stress significantly enhances animal resistance. Conversely, long-term high-intensity heat stress can cause damage to animals, mainly due to limb weakness, frequent drinking, increased sweating, incapability, and decreased central nervous system excitability. With the continuous warming of the global climate, combined with the increasing scale and stocking density of the breeding industry, the damage caused by heat stress to animals has become more serious and has become the most important stress-causing factor in southern China [2, 3]. For broilers, heat stress shows a decrease in feed intake, a decrease in feed conversion rate, and a slowing of the growth rate [5], while in laying hens, there is a decrease in the egg production rate, egg weight reduction, and eggs. The quality is reduced, and in severe cases, the death of laying hens can also be caused [6]. In the pig industry, heat stress causes damage to the reproductive performance of boars, which is manifested in decreased semen quality, decreased sperm density and sperm motility, and increased sperm deformity rate [7]. Sows have estrus and conception and abnormal growth of embryos [8]. It can be seen that heat stress has a serious impact on animal production performance. Therefore, it is of great significance to analyze the mechanism of heat stress and develop targeted prevention and control technology. Effects of heat stress on different body functions of animals are shown in Table 1.

### 2.4. Stress Causes Immune Dysregulation

Hyperthermia produces an extreme effect on livestock production [32]. Hyperthermia negatively affects animals' immune systems, making the animals more vulnerable to infections or diseases. There are two types of immune systems: adaptive and innate; both these systems interact and protect the body from harmful foreign agents. Heat stress disrupts the natural barrier to bacteria and may raise the endotoxin concentration that negatively affects vaccine bearing cells of the target [33]. Under stress conditions, the immune system and other body functions are adversely affected. Several stress hormones are produced by the HPA axis and sympathetic adrenal medullar (SAM) axis in response to stress. These stress hormones can induce changes in immune function by interacting with the receptors on immune cells. The difference in immune cells produces abnormalities in mouse normal functioning like sleeplessness, hyperthermia, less hunger, and desolation [34, 35].

### 2.5. Effects of Heat Stress on Immune Organs and Immune Cells

The immune system is a very complex system to investigate. Many researchers study various aspects of the immune system, but many elements are still not clear. Stress may affect the T cell number and functions of lymphoid organs. Many studies have indicated that heat stress reduces the weight of the thymus [52]. Studies have shown a marked change in the concentration of CD4 and CD8 cells at different temperatures [53]. High temperature causes an increase in the rate of apoptosis in mice [54]. Heat stress alters the T cell differentiation cycle that undergoes self-activation and is one of the causes of autoimmune diseases. Due to changes in the T cell pathway, the number of clones causes self-reactivity. These clones interfere with body normal immune functioning, so they cause diseases in the body [55]. Spleen and lymph nodes are affected by heat stress, and their weight may be reduced under heat stress conditions. The number of T cells in the spleen and lymph nodes increased with stress, but there are no detectable B cell changes [53]. A previous study clearly explains that heat stress shows marked structural variations in splenic parenchyma compared to the control group. These variations include lymphocytic necrosis and degeneration, especially at the periphery of lymphoid nodules with leukocyte infiltration. Moreover, substantial congested areas within the splenic red pulp were prominent. Cellular brownish pigments were observed along the congested blood vessels, which confirm hemosiderosis [34]. Cell-mediated immunity is an active response produced by antistimulator immune cells. The cells involved in cell-mediated immune responses are T lymphocytes and mononuclear cells, including NK cells, and granulocytes. Different cell subsets have different roles in cellular immunity. In vivo and in vitro experiments show that stress mainly inhibits cell-mediated immunity and manifests as thymus atrophy.

For the first time, the effect of heat stress on cell-mediated immune response was reported by Pitkin [35]. Chicken feeding under 36°C for five days caused a decrease in delayed type hypersensitivity and lymphocyte reactivity to decreased PHA. The effects of electrical stimulation of different intensities on cellular immune responses were observed systematically, and the transformation function of lymphocytes in whole blood was inhibited. And the inhibitory effect is proportional to the stress intensity [56]. Ocaña-Guzman et al. reported that stress could hinder the body's delayed hypersensitivity reaction and reduce T lymphocyte conversion function, which may be caused by endogenous opioids. Also, the stress-induced inhibition of T lymphocyte reaction may be related to the psychological state. It has also been reported that the phagocytic function of mononuclear macrophages in animals is weakened during the stress response. Cytotoxic T cell function also declined [57].

In mice during hyperthermia, the IgG, IgM, and antibody concentration and functioning of the humoral immune system are also reduced [38]. Hyperthermia also decreases lymphocyte count, antibody, and IgA secreting cells. In poultry, the activity of macrophages is also affected during heat stress. During heat stress in circulation, the number of heterophil and lymphocytes increases [37]. Heat stress produces reactive oxygen species in mice and Toll-like receptors stimulated under this environmental stress. TLRs are receptors located at the host-pathogen junction; they protect the host by recognizing any foreign material. Most of the pathogenic particles are detected by TLRs, which after passing through a series of activation stimulate cytokine release and affect the immunity [58].

Heat stress can significantly affect the immune function of the animal body. The study found that under heat stress conditions, the lymphocytes in the thymus and bursa of Fabricius were damaged in large numbers, and the development of lymphoid organs was blocked, which seriously damaged the body immune system [10]. Also, heat-stressed broilers showed significant reductions in IgM and IgG antibody levels in vivo [11]. The relationship between the hypothalamic-pituitary-adrenal (HPA) axis and the stress response is closely related. When the stress response occurs, the heat is transmitted to the hypothalamus, and the synthesis of corticotropin-releasing hormone (CRH) acts on the anterior pituitary to promote the synthesis and release of adrenocorticotropic hormone (ACTH). The released ACTH in turn activates the adrenocortical cells and eventually synthesizes and releases the glucocorticoid (GC). Studies have found that glucocorticoids have a significant regulatory consequence on the body immune system, and the release of excess GC inhibits the activity of immune cells, leading to further expansion of the body inflammation [16]. Koch et al. and other studies found that the secretion level of inflammatory factor IL-2 in the jejunum of pigs in the early stage of heat stress was significantly reduced. However, in the late stage of heat stress, the levels of IL-10 and IgA in jejunum tissues were significantly upregulated [12]. Pearce et al. reported that the content of IL-2 in the small intestine tissue of mice was significantly decreased in a high-temperature environment [59]. These studies have shown that heat stress can reduce the level of antibodies in animals and increase the expression of inflammatory factors, thereby causing serious damage to animal immune function.

### 2.6. Effects of Heat Stress on Inflammatory Cytokines

Recent studies have shown that excessive immune function is regulated by immunologically active cytokines. The inhibitory effect of stress on the immune system is also achieved by inhibiting immune-active cellular factors. Neuroendocrine response and immune-active cell production during stress multiply delivery qualities; there is a two-way regulatory activity between hormones and cells. Harbuz et al. reported that heat stress can suppress IL-1 and IL-2 production, interferon (INF), and tumor necrosis factor (TNF). Besides, there are reports of traumatic stress that can also reduce several immune-active cytokine productions. A certain degree of GC concentration increases during stress, simulating IL-1 action [60]. Several studies confirmed that stress also promotes the production of IL-4. Therefore, humoral immunity may have a certain promoting effect, while severe stress causes a destructive force and reduces IL-4 generation. IL plays a central role in the neuroendocrine response during stress and the immune system mutual regulation. It not only triggers an immune response but also has a direct effect on the central nervous system. This may cause fever, and it increases the release of adrenal cortex hormones, glucocorticoids, etc. *In vivo* and *in vitro* experiments showed that stress concentration of GC inhibited mouse peritoneal macrophages producing IL-1. It was found that the plasma of rats after heat injury can inhibit the secretion of spleen macrophage IL-1. It has been suggested that electroacupuncture stimulates the production of macrophage cells in the abdominal cavity. This may be due to the type of stress, time and intensity, animal species, and experimental conditions [61].

### 2.7. Effects of Heat Stress on GIT

Healthy GIT has a vital role in normal functioning, especially in the consumption and distribution of nutrients, water, and electrolyte balance and building of the mouse immune system [18]. The GIT protects the body from pathogenic microbes. Under unfavorable conditions, certain microbes enter the GIT and produce harmful effects and disturb the normal functioning of GIT. Some important factors that cause GIT abnormalities are contaminated food items, genetic effects, weather irregularities, and heat stress [57]. Under heat stress, all of these elements influence the GIT of the mouse and suppress the immune functioning and rupture the wall of GIT. This leads to an increase in host vulnerability towards many diseases and the rate of death [62]. Under normal conditions, the GIT absorbs the food particles by using its special receptors, which form a network with the cellular junctions. Under heat stress, these complex functions disrupt and inhibit the regular operation of the GIT barrier. The intestinal epithelium plays a crucial role in the protection of the body against infectious agents and toxins. Many factors (e.g., heat stress, endotoxin, and some drugs) affect this GI barrier and disturb its integrity [63]. Due to heat stress, the epithelium of GIT gets injured, and blood flow increases to protect the body from heat. This condition leads to ischemia, and it also increases epithelial permeability [64]. Ischemia of the intestine leads to the production of ROS. High levels of reactive oxygen species damage mouse protective systems and destroy genetic material, protein, and lipids [65].

The effects of high temperature on the mouse intestine have been investigated. These investigations have shown that many histological changes occur in the structure of the jejunum and ileum, and bleeding of villi is also evident. The permeability of the intestine increases after long-term exposure to heat stress [66]. In another study, during heat stress treatment after staining the small intestine, it was observed that the intestine walls get injured; sloughing of the head of villi and shedding of epithelium cells are also observed. Heat stress also impacts the length of intestinal villi. The cells of the upper part of the villi are disrupted and shed off during heat stress. The epithelial cells get detached from the lamina propria and are also spaced from each other. Moreover, the structures of mitochondria and endoplasmic reticulum are also affected. Heat stress treatment produces changes in the nucleus structure and enhances organelle in the lysosomes. Heat stress causes continuous disruption of epithelial cells from the membrane in the rat small intestine [67].

Figure 2 summarizes the effect of chronic heat stress on the intestinal mucosa. Chronic heat stress may enhance immune cell infiltration into lamina propria and muscularis mucosae of the intestine. At high-temperature bacterial compounds, pathogens and small particles like Lipopolysaccharides (LPS) may cause adaptive immune cell infiltration due to distorted intestinal barrier function. For example, LPS may enter the epithelial lining and stimulate the inflammatory response. Therefore, chronic heat stress may stimulate the intestine balancing mechanisms to maintain homeostasis between beneficial bacteria and the immune system [68].

High temperature causes marked disruption in reactive oxygen species and the production of antioxidants; this imbalance leads to harmful effects on a mouse body. Heat stress produces destruction and enhances apoptosis. The amount of MDA and ROS/RNS is enhanced in mouse small intestines (jejunum, ileum, and duodenum) under heat stress conditions. The SOD and GSH-px enzymes are involved in antioxidant activity during heat stress; their activity is decreased during the stress period. [69].

### 2.8. Effect on Intestinal Mucosal Barrier

As one of the body's largest digestive organs, the intestine is also the main storage place for microorganisms and endotoxins, and it is the first barrier to the body's nonspecific immunity. While digesting and absorbing various nutrients, a healthy and complete intestinal mucosal barrier can limit microorganisms and metabolites to a specific range in the intestine, preventing them from entering the blood circulation system and inducing epidemics [70]. According to the composition and function of the intestinal mucosal barrier of the animal body, the intestinal cavity to the mucosal layer is sequentially divided into a mechanical barrier, a chemical barrier, an immune barrier, and a biological barrier [71].

The tight connection between the mucus layer and mucosal epithelial cells forms a mechanical barrier in the intestine. Mucus secreted by goblet cells coats the surface of the intestinal epithelium to form a mucus layer, which can effectively prevent harmful substances such as bacteria and endotoxins from freely passing through the mucosal layer and entering the blood circulation system to damage the body [72]. Intestinal epithelial cells play a main role in maintaining the integrity of the mucosal barrier because it regulates the secretion of mucus and prevents endotoxins and bacteria from entering the submucosa freely [73]. Moreover, intestinal epithelial cells participate in the process of mucosal immunity by recognizing pathogenic bacteria, thereby regulating the activity of submucosal lymphocytes [74]. The connection structure between intestinal epithelial cells is composed of tight connection, gap connection, and adhesion connection. The structure between epithelial cells is based on tight junctions, which regulate the transport of substances between epithelial cells and thereby exert the permeability of the intestinal mucosal barrier. In addition, tight junctions play a role in the transmission of information between epithelial cells and the internal and external environment and play an important role in the maintenance of intestinal mucosal barrier function [75, 76]. As one of the largest mucosal immune organs in animals, the intestine plays a significant role in the functioning of the immune system. Intestinal mucosal lymphoid tissue, secreted antibodies, and cytokines in the intestine constitute the immune barrier of intestinal mucosa [75]. Intestinal mucosal cells ingest, process, and present antigens through pattern recognition receptors. Finally, T cells, B cells, and macrophages in the intestinal epithelium initiate the cellular immune process, thereby playing a role in protecting intestinal health. In production, the main means of treating inflammatory bowel disease are the use of antibiotics. Although it has a certain therapeutic effect, the excessive use of antibiotics can cause serious consequences, such as causing resistance in animals and breaking the intestinal tract. The microecological balance increases the risk of intestinal infections. In addition, drug residues in animals are another important issue that deserves attention [75]. The mucosal barrier formed by intestinal epithelial cells is a natural barrier for the body to absorb nutrients [77] and resist the invasion of pathogens (toxins) [78]. Its integrity is an important prerequisite for protecting the intestinal health of the host. Studies have shown that the integrity and permeability of intestinal epithelial cells mainly play a role through the tight connection between cells [71].

### 2.9. Effect of Heat Stress on Liver Functions

Heat stress produces deadly effects on living organisms. Heat stress induces a high rate of inflammatory reactions and oxidative stress. The increasing level of free radicals and inflammatory cytokines leads to a reduction in antioxidant species in the body that produces liver damage. Acute liver failure is related to heat stress; during heat stress, hypophosphatemia is identified in animals. Hyperthermia reduces hepatocyte expansion, enhances hepatocyte apoptosis, and promotes hepatocyte necrosis [79]. Under heat stress, the level of AST and ALT increases significantly. Heat induces structural alteration in hepatocytes and structural abnormality in the parenchyma of the liver. Glutathione peroxidase (GPX), malondialdehyde (MDA), and SODI levels were high. The amount of TNF-*α* was also increased during heat treatment in the liver [80].

### 2.10. Effect of Heat Stress on the Reproductive System

Heat stress affects the reproductive system of a mouse. Heat stress produces a disturbance in spermatogenesis, causes sperm cell destruction, and decreases fertility [81]. Heat stress negatively affects the reproduction system of animals and decreases the production rate. High temperatures produce alterations in the cellular functions of the reproductive organs [82]. Spermatogenesis is depending on temperature; high temperature can cause changes in this process. Heat stress has many side effects on the testes, like DNA aberrations in germ and sperm cells. Heat stress leads to decreased oocyte growth, embryonic maturation, placental growth, and decreased lactation. Spermatids and spermatocytes are mostly affected by heat stress [83]. Heat stress is a significant reason for DNA damage and apoptosis due to damage to spermatogenic cells. It has been reported that the growth of the embryo decreases the heat-stressed spermatozoon [76]. High temperature causes decreased luteinizing hormone release in both male and female reproductive systems [84]. Hyperthermia decreases gonadotropin receptor and aromatase activity of granulose cells in the animal. During the gestational period under heat stress, fetal development reduces. Fetal teratogenesis may also occur due to heat stress [77].

Heat stress decreases the oocyte competency, thus causing infertility in animals [26]. A study showed that chronic and acute heat stress reduces the ovary and gene expression of heat shock protein (HSP). Chronic heat stress decreased the whole body weight and ovarian development but had no significant effects on the ovarian index. In contrast, acute heat stress did not substantially impact entire body weight and ovarian growth. Acute and chronic heat stress equally disturbed the ovary function by dysfunctioning of granular cells. The previous study stated that the family member of HSP40, HSP70, and HSP90 was coexpressed to function after heat treatment in mice [85].

### 2.11. Activation of Mitogen-Activated Protein Kinase (MAPK) Pathway by Heat Stress

GIT can digest and absorb food particles through specific receptors. The cells of the epithelium are attached to the junction and form a network. Different junctions are present in the GIT that are adherent junction, tight junction, gap junction, and desmosomes; all are essential in transportation [67]. Many proteins are involved in maintaining the transportation and signaling pathways, including myosin light kinase (MLCK), mitogen-activated protein kinases (MAPKs), protein kinase C (PKC), PATJ, and small GTPases [78].

The MAPKs are a collection of essential threonine kinases produced under high temperatures by producing cytokines, ischemia, and ROS. MAPKs are stimulated under stress conditions and affect many cellular procedures like cell-mediated cell death, survival, adjustment, and cell multiplication [86]. ERK, c-Jun N-terminal kinases (JNK), and p38 MAPK are the three most important members of the family of MAPK. The MAPKs maintain the heat stress effects and also induce abnormalities in the epithelial cells. Adverse effects of heat stress are enhanced due to the inhibition of ERK1/2. At the same time, the intestinal epithelial cells are treated with the JNK or p38 MAPK inhibitors, reducing the negative effect of heat stress. A study's findings indicated that ERK1/2 acts as antiapoptosis, and JNK and p38 MAPK support apoptosis under heat stress in rat intestines [80].

### 2.12. Relation of Heat Stress to Tight Junction Proteins

Hyperthermia induces changes in tight junction proteins that can be predicted. It has been described by most researchers that hyperthermia enhances tight junction permeability. Studies have shown that tight junctions are mainly composed of structural and functional proteins. Structural proteins such as occludin, claudin family, and junctional adhesion molecules (JAM) constitute the structural skeleton. The ZO family is functional proteins in tight junction structures. Functional proteins, together with structural proteins and membrane proteins, play an important role in the maintenance of intestinal mucosal barrier function [81] and have become one of the hotspots of intestinal barrier function research in recent years. Studies indicate that constant exposure to high temperature causes upper regulation of occludin protein manifestation and decreases the flow of ZO-1. There is not any effect on the claudin-3 protein in Caco-2 cells [7]. There are 24 members of the claudin family, and they have different tasks. Claudin is divided into two groups: one group is involved in the development of a barrier, and the other is engaged in developing a channel. Claudin-2 reduces the rigidity of the epithelial barrier. Due to inflammation of the intestine, claudin-2 protein expression is increased [86]. Tight junction permeability is connected with the claudin expression. The level of TER increased due to overexpression of claudin; claudin-4 and claudin-2 reduced the level of TER. In mice with intestinal inflammation, the concentration of claudin-2 is higher than that of mice without intestinal inflammation. The study has reported that IL-6 boosts the tight junction permeability by increasing the expression of claudin-2 in the intestine's epithelial cells. IL-6 plays a crucial role in the maintenance of tight epithelial junctions of the intestine. IL-6 enhances the Cdx2 protein expression, whose activity is reduced by utilizing MEK and P13K suppression [87].

In mice, continuous introduction to high temperature leads to changes in the intestine's epithelial layer due to decreased length of villi and sloughing of the epithelium, so the inner layer lamina propria gets open to the elements. Frequent contact with high temperature induces changes in tight junction protein expression in the mouse. In animals, continuous exposure to hyperthermia causes the destruction of tight junctions, leading to the translocation of pathogens. These studies indicate that hyperthermia destroys the intestinal wall and produces changes in tight junction proteins, but the minuscule changes in tight junction protein appearance are under investigation [88].

### 2.13. Combating the Heat Stress in Animals

Heat stress is a significant environmental element in the context of global warming, and it has a negative impact on animal performance worldwide. High temperature during the summer period significantly lowers animal farming profitability [89]. Multidisciplinary approaches to heat stress protection are required, and these may include housing [90], genetics [91], heat conditioning, food, and nutrition [92]. According to Lin et al., there are a number of potential strategies for dealing with high ambient temperatures, including thermal conditioning and the intake of certain micronutrients, such as minerals and vitamins [93].

## 3. Conclusion

Heat stress produces harmful effects on mouse metabolism, reproductive system, immune system, and gut health. It is reported that hyperthermia enhances intestinal permeability and causes the destruction of the tight junction barrier. Further, endotoxemia and proinflammatory cytokines are also a contributor to the tight junction barrier in heat stress. It is concluded that heat stress lowers the body's metabolism, leading to a high mortality rate in animals. Several proteins are produced in response to heat stress, which shows that natural systems present that animals can survive in unfavorable conditions. Scientists are trying to understand different adaptation methods in animals' bodies to overcome the adverse effects of heat stress.

## Figures and Tables

**Figure 1:** Communication between the nervous and immune systems.

**Figure 2:** Effect of chronic heat stress on the intestinal mucosa.

**Table 1:** Effects of heat stress on different body functions of animals.

S.No	Species	Body functions involved	Effects of heat stress	References
1	Calves	Immune function	Decreased ratio of circulating antibodies (IgG and IgM), reduced systemic humoral responses, increased expression of inflammatory factors, effect on lactation performance, and damage to the immune function which ultimately affect the health and growth performance of calves	[12, 36–39]

2	Chickens	Gut function	Reduced nutrient absorption, poor performance of gut wall integrity, increased disease susceptibility, and higher mortality in chickens	[40]

3	Birds	Tight junction permeability	Compromised TJ barrier and luminal contents enter into the blood circulation. Therefore, a leaky gut induces chronic systemic inflammation which reduces the disease-resistance capacity of birds and induces changes in tight junction protein expression	[41, 42]

4	Birds and other animals	Reproductive function	Decreased secretion of the gonadotrophin-releasing hormone (GnRH) in laying birds which brings infertility and also delays in the process of ovulation via reducing follicular size, estradiol concentrations, and expression of LH receptors. Also effects on the epigenetic modification of sperms which interferes with the active demethylation of DNA in the male pronucleus of fertilized eggs, thereby reducing the fertility of sperms	[25, 43, 44]

5	Mice	Ovarian function	Heat stress damaged the ovary microstructures, thereby reducing fertility	[45]

6	Livestock	Growth and performance	Under HS, animals often have listlessness, shortness of breath, decreased food intake reducing growth performance, poor meat quality, reproductive performance, and immunity function which lead to death in severe cases	[46]

7	Pig/swine	Intestinal peristalsis	Under HS, the gastric emptying time and the intensity of intestinal peristalsis of animals are prolonged and weakened, which reduces the mechanical digestive function, resulting in accumulation of chyme and inhibition of appetite	[47]

8	Livestock and poultry rats	Intestinal absorption function	Serious damage to the intestinal structure by significant reduction of the height of intestinal villi, increase in the depth of crypt, decrease in the value of V/C, intestinal villi rupture, edema, and shedding of epithelial cells at the top of villi. Congestion, edema, exfoliation, and thinning of intestinal wall	[48–51]
